The article "Dynamic Rule-Based Algorithm to Tune Insulin-on-Board Constraints for a Hybrid Artificial Pancreas System" was published in 2020. Journal: J Healthc Eng.

# Dynamic Rule-Based Algorithm to Tune Insulin-on-Board Constraints for a Hybrid Artificial Pancreas System

**DOI:** 10.1155/2020/1414597

**Published:** 2020-01-11

**Authors:** Arthur Bertachi, Lyvia Biagi, Aleix Beneyto, Josep Vehí

**Affiliations:** ^1^University of Girona, Girona, Spain; ^2^Federal University of Technology–Paraná (UTFPR), Guarapuava, Brazil; ^3^Centro de Investigación Biomédica en Red de Diabetes y Enfermedades Metabólicas Asociadas, Madrid, Spain

## Abstract

The artificial pancreas (AP) is a system intended to control blood glucose levels through automated insulin infusion, reducing the burden of subjects with type 1 diabetes to manage their condition. To increase patients' safety, some systems limit the allowed amount of insulin active in the body, known as insulin-on-board (IOB). The safety auxiliary feedback element (SAFE) layer has been designed previously to avoid overreaction of the controller and thus avoiding hypoglycemia. In this work, a new method, so-called “dynamic rule-based algorithm,” is presented in order to adjust the limits of IOB in real time. The algorithm is an extension of a previously designed method which aimed to adjust the limits of IOB for a meal with 60 grams of carbohydrates (CHO). The proposed method is intended to be applied on hybrid AP systems during 24 h operation. It has been designed by combining two different strategies to set IOB limits for different situations: (1) fasting periods and (2) postprandial periods, regardless of the size of the meal. The UVa/Padova simulator is considered to assess the performance of the method, considering challenging scenarios. In silico results showed that the method is able to reduce the time spent in hypoglycemic range, improving patients' safety, which reveals the feasibility of the approach to be included in different control algorithms.

## 1. Introduction

Type 1 diabetes (T1D) is a chronic condition in which the pancreatic beta-cells either stop or reduce drastically the production of insulin. Insulin is a hormone whose function is to facilitate the glucose uptake from the bloodstream into the cells to be used or stored. Subjects with absence of insulin in the body face very high levels of blood glucose (BG) (hyperglycemia), which can lead to long-term micro- and macrovascular complications [1, 2]. Therefore, subjects living with T1D must inject insulin exogenously in order to regulate blood in a lifelong challenge [3], and intensive insulin therapy reduces the risk of long-term complications [4]. But maintaining blood glucose levels into near-normoglycemia is not a trivial task, and if insulin is overdosed, BG may fall to dangerously low levels (hypoglycemia), which can lead to serious hazards, such as diabetic coma or even death [5].

Over the last years, researchers have been working towards a closed-loop system to control BG automatically [6]. This system, known as artificial pancreas (AP), is usually composed of a continuous glucose monitor (CGM), a control algorithm, and continuous subcutaneous insulin infusion through a pump. Insulin-only AP systems consider only insulin infusion to control BG, and dual-hormone AP systems also consider glucagon infusion to elevate BG to reduce the risk of hypoglycemia. AP systems can also be classified into two different categories based on the degree of automation: hybrid closed-loop system, in which subjects are involved in the control loop and must announce meals or other disturbances to anticipate their effects, and fully closed-loop systems, where no actions are required from the patients [7, 8].

One of the main challenges of the AP system is achieving postprandial glucose control mainly because the insulin absorption through the subcutaneous tissue is slower than the appearance of glucose in the blood after a meal [9]. Due to this difference in dynamics of insulin action and carbohydrate (CHO) absorption, attempts to avoid hyperglycemic peaks are usually accompanied by hypoglycemic excursions [10]. Several approaches have been tested to overcome such issue [11–14], but while an ultrarapid insulin analogue is not available [15], postprandial control using subcutaneous route will continue to be a challenging situation for closed-loop systems. Diverse studies have included estimations of insulin concentration in the body to avoid excessive insulin stacking [16–19]; however, hypo- and hyperglycemia are still a hazard for AP systems, and novel approaches are still required.

Revert and colleagues introduced a safety auxiliary feedback element, so-called SAFE layer [20], to limit excessive insulin in the subcutaneous tissue, i.e., insulin-on-board (IOB). This layer is based on the sliding mode reference conditioning technique [21] and acts on the glucose reference signal when a specific constraint, related with the maximum IOB allowed ($\bar{\text{IOB}}$), is violated. Such technique has already been applied in different control schemes [22–25], but so far it is not clear the best methodology to tune $\bar{\text{IOB}}$. The selection of the constraint $\bar{\text{IOB}}$ is critical in the design of the closed-loop system. This parameter regulates insulin infusion based on an estimation of the IOB. As higher $\bar{\text{IOB}}$, more insulin the controller will be allowed to deliver. Considering that once insulin is injected into the body, it cannot be removed, it will act naturally lowering BG levels.

The Spanish Consortium on Artificial Pancreas and Diabetes Technology has been working over the last decade on the development of a new artificial pancreas system. In the first clinical trial, to evaluate the performance of the PD controller with the SAFE layer, an individualized constraint $\bar{\text{IOB}}$ was designed to control postprandial BG levels after the consumption of a meal with 60 grams of CHO [26]. The closed-loop controller achieved better outcomes compared with the open-loop therapy, reducing significantly the time spent in hyperglycemia without increase the risk of hypoglycemia. However, a limitation of this study is that $\bar{\text{IOB}}$ was tuned for this specific meal size. Therefore, novel approaches on how to select $\bar{\text{IOB}}$ for meals of different sizes are required to cope with daily-life operation of an AP system. In this work, a novel approach to tune $\bar{\text{IOB}}$ is presented. This new approach takes into account previous open-loop therapy to set $\bar{\text{IOB}}$ for periods without meals and in case of the announcement of meals, $\bar{\text{IOB}}$ can be raised to reduce hyperglycemia without leading to hypoglycemia in the late postprandial period. The proposal is evaluated in silico using the UVa/Padova simulator [27].

## 2. Materials and Methods

### 2.1. Control-Loop Scheme

In this section, the control scheme considered in this work is introduced. The control algorithm consists of two loops, as depicted by Figure 1. The inner loop is composed by a proportional derivative (PD) controller with an insulin feedback (IFB) loop. The outer loop contains the SAFE layer [20], which is inspired on the sliding mode reference conditioning technique [21]. This SAFE layer applies a discontinuous signal generated by a switching law when estimations of IOB ($\hat{\text{IOB}}$) surpass a preset limit of IOB ($\bar{\text{IOB}}$). Later, the discontinuous signal is filtered generating a smooth reference signal (*G*_rf_) to be applied into the controller. Therefore, this safety layer is able to maintain IOB inside desired bounds.

The control action produced by the PD controller is presented as follows:

(1) $$\begin{array}{c} u_{pd}\left(t\right)=K_{p}\left(\left(G_{\text{rf}}\left(t\right)-G\left(t\right)\right)+T_{d}\dot{G}\left(t\right)\right), \end{array}$$

where *K*_*p*_ is the proportional gain, *T*_*d*_ is the derivative time, *G*_rf_ is the glucose reference filtered after the action of the SAFE layer, and *G*(*t*) is the interstitial BG measurements provided by the CGM.

Then, the control action computed by the PD is augmented by two feed-forward signals: *u*_bolus_ and *u*_basal_. The signal *u*_basal_ is the insulin obtained from patients' daily basal profile. The term *u*_bolus_ is an impulse signal in case of the announcement of meals to compensate the disturbance caused by the ingestion of CHO.

The IFB algorithm [28] emulates the beta-cell physiology in healthy subjects, suppressing insulin secretion as plasma insulin concentration increases. The combination of the PD algorithm with both SAFE layer and IFB algorithm has already been investigated and shown to be more effective than when they are used separately [29]. The final control action signal provided to the insulin pump is

(2) $$\begin{array}{c} u_{d}\left(t\right)=u_{pd}\left(t\right)+u_{\text{basal}}\left(t\right)+u_{\text{bolus}}-\gamma {\hat{I}}_{p}\left(t\right), \end{array}$$

where *γ* is gain parameter and ${\hat{I}}_{p}$ is the is the estimated deviation of plasma insulin from steady state conditions (basal levels).

The term *G*_rf_ in equation (1) is the conditioned reference due to the action of the SAFE layer to maintain IOB below $\bar{\text{IOB}}$. Since the IOB is inaccessible, an insulin absorption model is considered to estimate IOB [30], through the following equation:

(3) $$\begin{array}{c} {\dot{C}}_{1}\left(t\right)=u_{d}\left(t\right)-K_{\text{DIA}}C_{1}\left(t\right),\\ {\dot{C}}_{2}\left(t\right)=K_{\text{DIA}}\left(C_{1}\left(t\right)-C_{2}\left(t\right)\right),\\ \hat{\text{IOB}}\left(t\right)=C_{1}\left(t\right)+C_{2}\left(t\right), \end{array}$$

where *C*_1_(*t*) and *C*_2_(*t*) are two compartments, *K*_DIA_ is a constant related with the duration of insulin action (DIA), and $\hat{\text{IOB}}$ is the estimation of IOB. The SAFE layer has a software-based nature and consists of two main elements: a switching block responsible to generate a discontinuous signal to maintain $\hat{\text{IOB}}$ into the desired range and a first-order filter to smooth the discontinuous signal before being applied to the main controller.

Consider the sliding function *σ*(*t*) defined by equation (4), the switching logic is defined as follows:

(4) $$\begin{array}{c} \sigma \left(t\right)=\hat{\text{IOB}}\left(t\right)-\bar{\text{IOB}}\left(t\right)+\tau \left(\dot{\hat{\text{IOB}}}\left(t\right)-\dot{\bar{\text{IOB}}}\left(t\right)\right), \end{array}$$

(5) $$\begin{array}{c} \omega \left(t\right)=\left\{\begin{array}{cc} W, & \text{if }\sigma \left(t\right)>0,\\ 0, & \text{otherwise,} \end{array}\right. \end{array}$$

with *W* > 0 mg/dl.

Finally, the discontinuous signal is filtered by the following equation and generates smooth changes in the glucose reference signal:

(6) $$\begin{array}{c} {\dot{G}}_{\text{rf}}\left(t\right)=-\lambda \left(G_{\text{rf}}\left(t\right)-G_{r}\left(t\right)+\omega \left(t\right)\right). \end{array}$$

Note that when *σ*(*t*) > 0, $\hat{\text{IOB}}$ is greater than $\bar{\text{IOB}}$. In order to drive $\hat{\text{IOB}}$ to the desired range, i.e., below $\bar{\text{IOB}}$, *u*_*d*_ must be decreased. The addition of *W* in equation (6) generates *G*_rf_ greater than *G*_*r*_, diminishing the insulin suggestion provided by the main controller and thus reducing $\hat{\text{IOB}}$. When $\hat{\text{IOB}}$ is below $\bar{\text{IOB}}$, no further action is provided by the outer loop, letting the controller work freely.

### 2.2. IOB Constraint Tuning

The selection of the constraint $\bar{\text{IOB}}$ is a critical point in the design of the control system. In this work, a new tuning approach for $\bar{\text{IOB}}$ is presented. In patients with T1D, insulin requirements vary during the day and also between days (intra- and interday variability). On traditional insulin pump therapy, physicians configure patients' pump to deliver a steady flow of basal insulin to cope with intraday variability. In addition, insulin boluses are delivered when meals are informed by patients, to cover the disturbance caused on glycemic balance due to the ingestion of CHO [3].

The artificial pancreas under development by our research group has been evaluated clinically, where 20 T1D subjects (age 40.7 ± 10.4 years, T1D duration 22.2 ± 9.9 years, and A1c 7.8 ± 0.7%) used the CL system in front of a mixed meal containing 60 grams of CHO [26]. In this trial, an individualized $\bar{\text{IOB}}$ tune was considered in order the improve postprandial glycemic control when compared with standard open-loop therapy. For this specific trial, where a single meal with 60 grams of CHO was consumed, $\bar{\text{IOB}}$ was adjusted based on parameters taken from patients' open-loop therapy and computed in an offline procedure. The procedure to compute $\bar{\text{IOB}}$ was as follows: considering that patients were in basal levels of IOB, $\bar{\text{IOB}}$ was computed as the estimation of IOB levels 90 minutes after the administration of an augmented bolus, by equation (3), to compensate this 60 grams meal. This augmented bolus was computed by adding to the standard bolus the amount of basal insulin that would have been delivered in the next hour in the case of being in open-loop therapy. Therefore, knowing in advance the size of the meal and all the parameters necessary to compute this augmented bolus, it was possible to compute in an offline fashion what would be the estimation of IOB levels 90 minutes after the meal bolus. This single value was applied as IOB limit during in this clinical trial [26].

Due to the huge amount of insulin in meal boluses, $\hat{\text{IOB}}$ violates $\bar{\text{IOB}}$, and a high frequency discontinuous signal is generated by the SAFE layer in order to return $\hat{\text{IOB}}$ back to $\bar{\text{IOB}}$ bounds. This action forces insulin delivery to zero for approximately 90 minutes, minimizing the effects of controller's overcorrection. When *σ*(*t*) ≤ 0 (equation (4)), insulin infusion may be restored if the controller deems necessary.

However, a single value of $\bar{\text{IOB}}$ may not be sufficient for 24-hour operation, especially due to the large intrapatient variability in T1D and to the different activities performed by subjects in their daily-life. The major problem observed in the strategy presented previously is that too high values of $\bar{\text{IOB}}$ may cause that the SAFE layer be ineffective because it will act in very few conditions, e.g., only after a meal bolus. It is comprehensible having higher $\bar{\text{IOB}}$ tuning during postprandial periods, especially because subjects tend to underestimate the CHO content in meals [31]. However, during late postprandial period, where the effects of meals have been covered either by the bolus or by the controller suggestions, such high values of $\bar{\text{IOB}}$ may lead to excess of insulin in the body, increasing the risk of hypoglycemia.

In this work, a new method to tune $\bar{\text{IOB}}$ to overcome the limitations presented by the former strategy is proposed. The new approach is called “dynamic rule-based” (DRB) algorithm and is intended to be used on hybrid artificial pancreas systems for 24-hour operation, where meals of any size are consumed. The proposed approach combines two different strategies to set $\bar{\text{IOB}}$ for different situations: (1) fasting periods: where no big disturbance is expected, and the controller must deal mainly with intraday variability and (2) postprandial periods: where a substantial raise in BG levels is expected due to the consumption of a meal and insulin bolus may not be enough to compensate such disturbance. In summary, the DRB algorithm generates a time-varying $\bar{\text{IOB}}$ based on patients' basal insulin profile taken from open-loop therapy, and when a meal is announced, the algorithm evaluated in real-time if $\bar{\text{IOB}}$ should be increased temporarily in order to reduce hyperglycemia. The following sections depict the algorithm, and a flowchart is also presented in Figure 2 to clarify the operation of the DRB algorithm.

#### 2.2.1. Fasting Periods

During fasting period (sleeping hours or daytime fasting periods), the absence of external disturbances makes the intraday variability the major challenge for the controller. The basal insulin profile from patients' open-loop therapy is considered to create a baseline for $\bar{\text{IOB}}$:

(7) $$\begin{array}{c} {\bar{\text{IOB}}}_{\text{bl}}\left(t\right)=K_{\text{IOB}}\left(\frac{2\cdot u_{\text{basal}}\left(t\right)}{60\cdot K_{\text{DIA}}}\right), \end{array}$$

where ${\bar{\text{IOB}}}_{\text{bl}}$ is the baseline for $\bar{\text{IOB}}$ and *K*_IOB_ is a gain that regulates the amplitude of ${\bar{\text{IOB}}}_{\text{bl}}$, with *K*_IOB_ > 0. In case of *K*_IOB_ < 1, $\hat{\text{IOB}}$ will not be allowed to be greater than it would have been during open-loop therapy. On the contrary, with *K*_IOB_ > 1, the insulin controller can suggest more insulin than what is programmed by the open-loop therapy. Thus, *K*_IOB_ should be selected in order to protect patients from hypoglycemia but also allowing the control algorithm to suggest insulin above open-loop regimen when necessary. Thus, during fasting periods, $\bar{\text{IOB}}$ is set to be equal to ${\bar{\text{IOB}}}_{\text{bl}}$. In this work, the parameter *K*_IOB_ is set to 1.3 for daytime period (06:00–23:00) and to 1.1 for night-time period (23:00–06:00).

Although this approach may be able to provide good glycemic control in front of intraday variability, patients in free-living conditions take CHO on several occasions during the day, requiring a greater amount of insulin for these periods. Therefore, the strategy of $\bar{\text{IOB}}$ during fasting periods is combined with another one, intended for postprandial periods, presented in the following section.

#### 2.2.2. Postprandial Periods

The tuning of $\bar{\text{IOB}}$ during postprandial period is an extension to the method already validated clinically by Rossetti and colleagues [26]. Here, the method is generalized for meals with different amount of CHO and also includes a set of rules based on BG readings to modify $\bar{\text{IOB}}$. This set of rules has been designed to determine if it is necessary to increase $\bar{\text{IOB}}$, for cases which the bolus was not enough to drive BG to near-normoglycemia levels.

The method works as follows: in case of the announcement of a meal, an insulin bolus is delivered as a feed-forward action. This bolus is an augmented version of the standard bolus computation, by adding a portion of the future basal delivery according to the size of the meal, as shown in the following equation:

(8) $$\begin{array}{c} u_{\text{bolus}}=\frac{M_{\text{CHO}}}{I2C}+\frac{G\left(t\right)-G_{r}}{\text{CF}}\;+\;\left(\int_{t}^{t+M_{\text{CHO}}}u_{\text{basal}}\left(t\right)\right)\frac{M_{\text{CHO}}}{60}, \end{array}$$

where *M*_CHO_ is the content of CHO of the meal (in grams), *I*2*C* is the insulin-to-CHO ratio, *G*_*r*_ is the BG reference, and CF is the correction factor.

After the bolus, $\hat{\text{IOB}}$ surpasses $\bar{\text{IOB}}$, and then *u*_final_ is forced to zero, while $\hat{\text{IOB}}$ is greater than $\bar{\text{IOB}}$, due to the action of the SAFE layer. The parameter *T*_IOB_ (in minutes, equation (9)) is introduced to regulate the starting time after the meal from when $\bar{\text{IOB}}$ may be increased. After *T*_IOB_ minutes, BG readings start to be evaluated in order to check whether $\bar{\text{IOB}}$ needs to be increased, aiming to drive BG below a selected target ($\underline{G}$). If in this moment, BG is greater than a threshold ($\bar{G}$), a new IOB limit is computed to control postprandial BG, based on equation (10). This value is maintained as $\bar{\text{IOB}}$, while BG is greater than $\underline{G}$. Finally, when BG returns to values below $\underline{G}$, $\bar{\text{IOB}}$ returns to follow ${\bar{\text{IOB}}}_{\text{bl}}$. Note that the parameters $\underline{G}$ and $\bar{G}$ can be adjusted intuitively by physicians. For a more aggressive postprandial control, these parameters should be decreased as follows:

(9) $$\begin{array}{c} T_{\text{IOB}}=1.5\cdot M_{\text{CHO}}, \end{array}$$

(10) $$\begin{array}{c} {\bar{\text{IOB}}}_{\text{PP}}=\max\left(\hat{\text{IOB}}\left(t-1\right),{\bar{\text{IOB}}}_{\text{bl}}\left(t\right)\right). \end{array}$$

The final tuning for $\bar{\text{IOB}}$ is determined during a real-time procedure, based on the dynamic behavior of patients basal insulin profile and also in the set of rules activated after the announcement of meals, to increase $\bar{\text{IOB}}$ during postprandial periods. Figure 2 depicts a flowchart of the proposed method to facilitate the understanding.

The variables “PP_state” and “flag_PP” included in Figure 2 were considered for implementation purposes. In the initialization of the system, both variables should be set to zero. “PP_state” indicates that a meal has been consumed, and that $\bar{\text{IOB}}$ may be increased considering a set of rules to evaluated BG levels *T*_IOB_ minutes after the announcement of the meal. The variable “flag_PP” guarantees that a single value of ${\bar{\text{IOB}}}_{\text{PP}}$ is computed for each meal.  Figure 3 depicts the application of the method in one representative virtual patient during a simulation, with a meal containing 45 g of CHO at 07:30 (represented by the green triangle in Figure 3(a)). Note that 67.5 minutes after the meal (computed by equation (9)), the limit of IOB has been increased because BG levels were above $\bar{G}$. When $\bar{\text{IOB}}$ was increased, the controller suggested more insulin in order to reduce the postprandial excursions since the insulin bolus was not enough for this specific meal. This period of time represents the first meal of a single patient during Scenario C, which is detailed in Section 2.3.3.

In summary, the DRB algorithm has been designed to make use of patients' basal profile, which is an indicative of insulin requirements along the day, combined with a modified version of the approach already tested clinically with real patients, which achieved good results during postprandial control. In addition, BG measurements has been incorporated to set $\bar{\text{IOB}}$, aiming to track glucose back to regular values safely. All the relevant parameters used in the simulations are listed in Table 1.

### 2.3. In Silico Evaluation

The proposed method is validated in the UVa/Padova simulator [27] on three challenging scenarios, including intrapatient variability in insulin sensitivity and in meal absorption rate [32].

Circadian variability has been included to simulate different requirements of insulin during the day and follows a sinusoidal variation. The parameters *V*_*mx*_ and *k*_*p*3_, which are related with the insulin sensitivity are modified as follows:

(11) $$\begin{array}{c} q\left(t\right)=q_{0}+0.3\cdot q_{0}\cdot \;\sin\left(\frac{2\pi }{24\cdot 60}\right)t+2\pi \cdot \text{rand}, \end{array}$$

where *q*(*t*) is the corresponding time-varying parameter; *q*_0_ is the default individual parameter value (*V*_*mx*_ or *k*_*p*3_), and rand is a uniformly distributed random number between 0 and 1.

Additionally, meal absorption rate and insulin absorption parameters (parameters *k*_*abs*_, *k*_*d*_, *k*_*a*1_, and *k*_*a*2_) assume different values (±30% around the standard value) after every single meal consumption. Further details about the aforementioned parameters are described elsewhere [27, 33].

#### 2.3.1. Scenario A

This scenario is considered to compare the performance of the DRB algorithm (${\bar{\text{IOB}}}_{\text{DRB}}$) against the method already validated clinically, with a fixed value for $\bar{\text{IOB}}$ (${\bar{\text{IOB}}}_{F}$). In a 7-day scenario, the adult cohort consumed a single meal containing 60 grams of CHO per day, between 10:00 and 16:00, in order to assess the postprandial control under different intrapatient variability conditions. This amount of CHO has been selected to conduct a fairly comparison since the former strategy was clinically validated for this specific meal size.

#### 2.3.2. Scenario B

This scenario is considered to compare the performance of the DRB algorithm (${\bar{\text{IOB}}}_{\text{DRB}}$) in front of meals with CHO content varying between 40 and 120 grams of CHO. In a 45-day scenario, the adult cohort consumed a single meal per day, between 08:00 and 19:00, in order to assess the postprandial control under different intrapatient variability conditions. It is considered just a single meal per day in order to avoid the accumulated effects of meals in the results.

#### 2.3.3. Scenario C

A 14-day scenario is considered to assess the performance of the proposed method intended to mimic real-life operation of the AP systems. A total of three meals, with different amounts of CHO, are consumed per day at 7:30 (45 grams), 13:00 (90 grams), and 18:30 (50 grams). An error of ±15% on CHO counting has also been included to challenge the system. To apply meal absorption variability, the 10 mixed meal models from each patient were randomly assigned for each meal intake along with the simulation. A total of four different strategies are applied in this scenario: (1) the DRB algorithm to adjust $\bar{\text{IOB}}$ (${\bar{\text{IOB}}}_{\text{DRB}}$), (2) a fixed value of $\bar{\text{IOB}}$ as used in Scenario A (${\bar{\text{IOB}}}_{F}$), (3) $\bar{\text{IOB}}$ is set to be equal to ${\bar{\text{IOB}}}_{\text{bl}}$, without the rules considered for postprandial period (${\bar{\text{IOB}}}_{\text{bl}}$), and (4) the same insulin controller considered in other strategies, but without $\bar{\text{IOB}}$.

## 3. Results and Discussion

In this section, glycemic outcomes are presented for all the scenarios previously described. The performance of different methods to adjust $\bar{\text{IOB}}$ is evaluated according the time spent into different glycemic ranges [34]. Results are computed based on CGM measurements. Individual metrics for the adult cohort from the simulator are computed, and then the results are presented as the median (25th–75th percentile) among the cohort. Additionally, the occurrence of hypoglycemic episodes (defined as at least 15 consecutive minutes with glucose below 70 mg/dl) is also analyzed.

### 3.1. Scenario A

Table 2 shows the metrics for Scenario A. These metrics assess the performance of ${\bar{\text{IOB}}}_{\text{DRB}}$ and ${\bar{\text{IOB}}}_{F}$ during postprandial period (i.e., 4 hours following the meal), once the last has been designed for such purpose. The metrics used for this evaluation are: average BG levels, percentage of time spent in different glycemic ranges, glycemic excursion (defined as the difference between the maximum BG level and the premeal BG level), and the total insulin delivered by the controller after the meal bolus.

Note that both strategies achieved similar results. Although ${\bar{\text{IOB}}}_{F}$ obtained numerical results slightly superior than the proposed method, no significant difference was observed in any of the metrics. The new strategy (${\bar{\text{IOB}}}_{\text{DRB}}$), besides being applicable for meals of any size, achieved equivalent outcomes when compared with the former strategy, which was designed for meals with 60 grams of CHO and achieved good results in real patients.

However, analyzing the whole simulation period (7-days), the new strategy was able to eliminate the occurrence of hypoglycemic events, while five events were observed for ${\bar{\text{IOB}}}_{F}$. This fact reinforces the hypothesis that modifying $\bar{\text{IOB}}$ over the day increases patients safety.

### 3.2. Scenario B

Table 3 shows the metrics during postprandial period in Scenario B for the two methods applied in this Scenario B.

Different from Scenario A, in Scenario B, meals from different sizes were considered to evaluate the postprandial performance of the controller, which is more realistic. Results showed a slight superiority of the ${\bar{\text{IOB}}}_{\text{DRB}}$ against the ${\bar{\text{IOB}}}_{F}$ in all the glycemic metrics analyzed. Notice that the percentage of time spent in tight glycemic range increased from 38.1% to 41.52%, while the percentage of time spent in hyperglycemia reduces at the same time, from 15.63% to 14.14%. This analysis shows that the previous tuning of $\bar{\text{IOB}}$ may not be sufficient for varied size of meals.

### 3.3. Scenario C

Table 4 shows the results for the 14-day scenario comparing the system with the DRB algorithm (${\bar{\text{IOB}}}_{\text{DRB}}$) against the other strategies. It displays the mean glucose, percentage of time spent in different glycemic ranges and the number of hypoglycemic events for the entire cohort.

The results display the solid performance of the strategies using the SAFE layer when compared with the insulin controller without IOB limitation, mainly to avoid hypoglycemia. The arm with the ${\bar{\text{IOB}}}_{\text{DRB}}$ strategy achieved the lowest amount of hypoglycemic events when compared with the other methods. The ${\bar{\text{IOB}}}_{F}$ strategy is the one with the lowest mean glucose values during daytime, but the fixed value of $\bar{\text{IOB}}$ is not enough to avoid hypoglycemic events, especially during night-time. On the contrary, the ${\bar{\text{IOB}}}_{\text{bl}}$ arm considered only the adjustment for $\bar{\text{IOB}}$ presented in Section 2.2.1. Such approach did not consider the rule-based algorithm to increase $\bar{\text{IOB}}$ during postprandial periods, and this is reflected in the slightly worse outcomes for this strategy when compared with ${\bar{\text{IOB}}}_{\text{DRB}}$, during daytime. The ${\bar{\text{IOB}}}_{\text{DRB}}$ arm achieved lower mean glucose values and spent less time in the hyperglycemic range, when compared with the ${\bar{\text{IOB}}}_{\text{bl}}$ arm.

Also during daytime, it can be observed that ${\bar{\text{IOB}}}_{\text{DRB}}$ achieved higher mean glucose values when compared with the insulin controller without $\bar{\text{IOB}}$, considerably above the *G*_*r*_. Although these values are higher than in healthy people, they are still acceptable considering the recommendations of the American Diabetes Association (ADA) [35], which is A1C <7% for nonpregnant adults. The median GMI (glucose management indicator) achieved by the proposed method during daytime is 6.7%, which gives the approximate A1C levels based on CGM measurements [36]. During night-time, ${\bar{\text{IOB}}}_{\text{DRB}}$ was able to lower mean glucose, without any hypoglycemic event. Considering 24-hour period for the entire scenario, the proposed method achieved a median GMI of 6.5%, within the limits recommendable by the ADA.

The control-variability grid-analysis (CVGA) [37], in Figure 4, allows a graphical visualization regarding the glycemic variability within an observational period of 24 hours. Note that the ${\bar{\text{IOB}}}_{\text{DRB}}$ approach achieved the highest percentage of points falling either in Zone A or Zone B, with 97.85%. Additionally, Figure 5 shows the dynamics of BG and insulin delivery for a single day, comparing ${\bar{\text{IOB}}}_{\text{DRB}}$ with the arm without IOB limits, to better illustrate the influence of the $\bar{\text{IOB}}$ in the control action.

Observing the results in Table 4 and Figure 4 it is possible to note that the action of the SAFE layer avoids the overreaction of the insulin controller due to the rise of glucose, caused by the meals. Although the results obtained by the DRB algorithm are only slightly better when compared with the other strategies which included the SAFE layer, it was observed a reduction on the occurrence of hypoglycemic events without leading to excessive hyperglycemia. All the three hypoglycemic events observed in the ${\bar{\text{IOB}}}_{\text{DRB}}$ arm were caused by the meal bolus and not by any insulin suggested by the controller after the meal. Therefore, the hypoglycemic episodes were very likely caused by overestimation of CHO content to compute the bolus.

The starting point of the proposed method was another strategy which has already been extensively tested both in silico and clinically, making the task of achieving better results even more difficult. Nevertheless, it has been possible to improve slightly the performance of the AP system in this in silico study, being able to apply different limits of IOB according to the CHO content of meals and by applying a lower $\bar{\text{IOB}}$ during night-time. Any improvement in postprandial glycemic control can reflect in a reduction on the risks associated with long-term complications, given its correlation with A1C levels [38], and the avoidance of nocturnal hypoglycemia is a major concern in T1D treatment. In addition, it also allows modification on the parameters of the proposed algorithm to be performed intuitively by physicians, if they deem necessary to further improvements on glycemic control. However, clinical trials involving real patients must be conducted to assess the performance of the proposed algorithm under real-life operation, in which patients may forget to announce meals, and the performance of the DRB algorithm may not be suitable to avoid hyperglycemia. Furthermore, the DRB algorithm may not be applicable in fully automatic AP systems, in which patients do not need to announce meals. Finally, the adjustments of $\bar{\text{IOB}}$ is a major task for AP systems which considers the SAFE layer, and the proper adjustment of this constraint also plays an important role even during physical activity [39, 40], by reducing the amount of injected insulin during and after exercise.

## 4. Conclusions

The dynamic rule-based algorithm proposed in this work has been designed to tune in real-time limiting of IOB to safely control BG levels. This algorithm is intended for 24-hour operation, which includes postprandial and fasting periods. During postprandial periods, it allows the increase of IOB limits when more insulin is required to have a more aggressive controller but yet safe. The strategy has been evaluated in silico under challenging conditions and achieved satisfactory performance, with emphasis on the reduction of hypoglycemic events during nocturnal period and without excessive hyperglycemia during postprandial period for meals with different CHO contents. Although, in this paper, the proposed strategy has been applied and evaluated in a PD controller, such approach could also be used by other algorithms, since the SAFE layer can be added to control algorithms of any nature.

## Figures and Tables

**Figure 1:** Control scheme based on a PD controller with IFB and with the SAFE layer. PK, pharmacokinetic.

**Figure 2:** Flowchart describing how the proposed dynamic rule-based algorithm works.

**Figure 3:** Operation of the dynamic rule-based algorithm during a postprandial period. Note that, after the meal (consumed at 07:30 and represented by the green triangle), the algorithm deemed necessary to increase $\bar{\text{IOB}}$ because BG levels were above $\bar{G}$. (a) BG measurements in mg/dl. (b) Insulin delivery. (c) The conditioned reference signal *G*_rf_. (d) Estimation of IOB levels and the constraint $\bar{\text{IOB}}$.

**Figure 4:** Control-variability grid-analysis for different arms evaluated in scenario C: (a) ${\bar{\text{IOB}}}_{\text{DRB}}$, (b) ${\bar{\text{IOB}}}_{F}$, (c) ${\bar{\text{IOB}}}_{\text{bl}}$, and (d) without $\bar{\text{IOB}}$.

**Figure 5:** Comparison of the dynamics of BG and insulin delivery between the controller with the DRB algorithm and without $\bar{\text{IOB}}$ for a single patient in scenario C: (a) BG readings; (b) insulin delivery.

**Table 1:** Parameters considered in this work for both inner and outer loops.

Parameter	Value	Unit
*K*_*p*_	TDI/2250	*U*/min
*T*_*d*_	90	min
*G*_*r*_	100	md/dl
*Γ*	0.42	*L*/min
*W*	350	mg/dl
*Τ*	10	min
*Λ*	0.1	min
*K*_DIA_	0.013	min^−1^
$\bar{G}$	150	mg/dl
$\underline{G}$	140	mg/dl

TDI, total daily insulin.

**Table 2:** Population metrics for postprandial glycemic control in scenario A.

	Mean glucose	Percentage of time spent in				Excursion (mg/dl)	Total basal (U)
	(mg/dl)	70–140	70–180	>180	<70		
${\bar{\text{IOB}}}_{\text{DRB}}$	141.48	46.58	96.13	3.87	0.00	62.00	3.56
	(136.4–153.0)	(24.7–56.5)	(93.8–100.0)	(0.0–6.3)	(0.0–0.0)	(55.9–67.3)	(3.0–4.0)

${\bar{\text{IOB}}}_{F}$	141.40	47.77	96.43	3.57	0.00	63.36	3.78
	(136.7–150.8)	(25.6–53.6)	(94.0–100.0)	(0.0–6.0)	(0.0–0.0)	(53.6–68.7)	(3.1–4.1)

**Table 3:** Population metrics for postprandial glycemic control in scenario B.

	Mean glucose	Percentage of time spent in				Excursion (mg/dl)	Total basal (U)
	(mg/dl)	70–140	70–180	>180	<70		
${\bar{\text{IOB}}}_{\text{DRB}}$	146.79	41.52	85.86	14.14	0.00	71.79	3.19
	(144.7–154.7)	(35.4–48.5)	(77.7–90.2)	(9.8–20.8)	(0.0–0.0)	(66.1–74.7)	(2.1–3.6)

${\bar{\text{IOB}}}_{F}$	148.96	38.10	84.38	15.63	0.00	75.43	3.43
	(147.0–156.2)	(25.3–47.3)	(77.1–86.3)	(13.7–22.9)	(0.0–0.0)	(69.0–79.4)	(2.6–4.1)

**Table 4:** Population metrics comparing the performance of the system with the dynamic rule-based algorithm (${\bar{\text{IOB}}}_{\text{DRB}}$) against other strategies, in scenario C.

	${\bar{\text{IOB}}}_{\text{DRB}}$	${\bar{\text{IOB}}}_{F}$	${\bar{\text{IOB}}}_{\text{bl}}$	Without $\bar{\text{IOB}}$
Daytime (06:00–23:00)				
Mean glucose	140.30 (134.2–143.5)	135.57 (133.0–140.3)	142.72 (134.7–145.3)	116.92 (114.0–121.6)
% of time spent in				
70–140	56.58 (49.3–66.3)	60.17 (56.1–65.4)	53.43 (46.3–64.6)	71.53 (67.4–79.4)
70–180	92.10 (85.5–95.3)	92.70 (85.9–96.6)	90.91 (85.2–95.0)	90.88 (83.5–93.7)
>180	7.90 (4.7–14.5)	7.30 (3.4–14.1)	9.09 (5.0–14.8)	5.25 (3.0–8.4)
<70	0.00 (0.0–0.0)	0.00 (0.0–0.0)	0.00 (0.0–0.0)	5.27 (0.4–9.9)
<54	0.00 (0.0–0.0)	0.00 (0.0–0.0)	0.00 (0.0–0.0)	1.61 (0.0–6.3)
# Hypoglycemic events	3	4	4	112
Night-time (06:00–23:00)				
Mean glucose	114.61 (112.1–118.8)	106.51 (104.0–107.2)	114.81 (112.9–126.1)	102.37 (100.1–103.9)
% of time spent in				
70–140	98.09 (94.3–99.1)	99.36 (96.0–100.0)	97.75 (87.2–99.2)	98.04 (96.0–99.3)
70–180	100.00 (100.0–100.0)	100.00 (100.0–100.0)	100.00 (100.0–100.0)	98.13 (97.1–99.4)
>180	0.00 (0.0–0.0)	0.00 (0.0–0.0)	0.00 (0.0–0.0)	0.00 (0.0–0.0)
<70	0.00 (0.0–0.0)	0.00 (0.0–0.0)	0.00 (0.0–0.0)	1.87 (0.6–2.9)
<54	0.00 (0.0–0.0)	0.00 (0.0–0.0)	0.00 (0.0–0.0)	0.13 (0.0–0.9)
# Hypoglycemic events	0	4	0	11

## Data Availability

The data used to support the findings of this study are available from the corresponding author upon request.

## Abbreviations

ADA: American Diabetes Association
AP: Artificial pancreas
BG: Blood glucose
CGM: Continuous glucose monitor
CHO: Carbohydrates
DIA: Duration of insulin action
DRB: Dynamic rule-based
IFB: Insulin feedback
IOB: Insulin-on-board
PD: Proportional derivative
PK: Pharmacokinetic
SAFE: Safe auxiliary feedback element
T1D: Type 1 diabetes.

## References

[1] Lind M., Svensson A.-M., Kosiborod M. (2014). Glycemic control and excess mortality in type 1 diabetes. *New England Journal of Medicine*.

[2] Zaccardi F., Webb D. R., Yates T., Davies M. J. (2016). Pathophysiology of type 1 and type 2 diabetes mellitus: a 90-year perspective. *Postgraduate Medical Journal*.

[3] Walsh J., Roberts R., Varma C., Bailey T. (2003). *Using Insulin: Everything You Need for Success with Insulin*.

[4] Nathan D. M., DCCT/EDIC Research Group (2014). The diabetes control and complications trial/epidemiology of diabetes interventions and complications study at 30 years: Overview. *Diabetes Care*.

[5] Graveling A. J., Frier B. M. (2017). The risks of nocturnal hypoglycaemia in insulin-treated diabetes. *Diabetes Research and Clinical Practice*.

[6] Bekiari E., Kitsios K., Thabit H. (2018). Artificial pancreas treatment for outpatients with type 1 diabetes: systematic review and meta-analysis. *BMJ*.

[7] Thabit H., Hovorka R. (2016). Coming of age: the artificial pancreas for type 1 diabetes. *Diabetologia*.

[8] Doyle F. J., Huyett L. M., Lee J. B., Zisser H. C., Dassau E. (2014). Closed-loop artificial pancreas systems: engineering the algorithms. *Diabetes Care*.

[9] Gingras V., Taleb N., Roy-Fleming A., Legault L., Rabasa-Lhoret R. (2018). The challenges of achieving postprandial glucose control using closed-loop systems in patients with type 1 diabetes. *Diabetes, Obesity and Metabolism*.

[10] Goodwin G. C., Medioli A. M., Carrasco D. S., King B. R., Fu Y. (2015). A fundamental control limitation for linear positive systems with application to type 1 diabetes treatment. *Automatica*.

[11] Luijf Y. M., van Bon A. C., Hoekstra J. B., DeVries J. H. (2010). Premeal injection of rapid-acting insulin reduces postprandial glycemic excursions in type 1 diabetes. *Diabetes Care*.

[12] Rossetti P., Ampudia-Blasco F. J., Laguna A. (2012). Evaluation of a novel continuous glucose monitoring-based method for mealtime insulin dosing-the iBolus-in subjects with type 1 diabetes using continuous subcutaneous insulin infusion therapy: a randomized controlled trial. *Diabetes Technology & Therapeutics*.

[13] Reddy M., Pesl P., Xenou M. (2016). Clinical safety and feasibility of the advanced bolus calculator for type 1 diabetes based on case-based reasoning: a 6-week nonrandomized single-arm pilot study. *Diabetes Technology & Therapeutics*.

[14] Turksoy K., Hajizadeh I., Samadi S. (2017). Real-time insulin bolusing for unannounced meals with artificial pancreas. *Control Engineering Practice*.

[15] Al-Tabakha M. M. (2015). Future prospect of insulin inhalation for diabetic patients: the case of afrezza versus exubera. *Journal of Controlled Release*.

[16] Ellingsen C., Dassau E., Zisser H. (2009). Safety constraints in an artificial pancreatic *β* cell: an implementation of model predictive control with insulin on board. *Journal of Diabetes Science and Technology*.

[17] Hajizadeh I., Rashid M., Samadi S. (2018). Adaptive and personalized plasma insulin concentration estimation for artificial pancreas systems. *Journal of Diabetes Science and Technology*.

[18] Toffanin C., Zisser H., Doyle F. J., Dassau E. (2013). Dynamic insulin on board: incorporation of circadian insulin sensitivity variation. *Journal of Diabetes Science and Technology*.

[19] Hajizadeh I., Rashid M., Turksoy K. (2017). Plasma insulin estimation in people with type 1 diabetes mellitus. *Industrial & Engineering Chemistry Research*.

[20] Revert A., Garelli F., Pico J. (2013). Safety auxiliary feedback element for the artificial pancreas in type 1 diabetes. *IEEE Transactions on Biomedical Engineering*.

[21] Garelli F., Mantz R. J., Battista H. D. (2011). *Advanced Control for Constrained Processes and Systems*.

[22] León-Vargas F., Garelli F., De Battista H., Vehí J. (2015). Postprandial response improvement via safety layer in closed-loop blood glucose controllers. *Biomedical Signal Processing and Control*.

[23] Hu R., Li C. (2015). An improved PID algorithm based on insulin-on-board estimate for blood glucose control with type 1 diabetes. *Computational and Mathematical Methods in Medicine*.

[24] Sánchez-Peña R., Colmegna P., Garelli F. (2018). Artificial pancreas: clinical study in Latin America without premeal insulin boluses. *Journal of Diabetes Science and Technology*.

[25] León-Vargas F., Garelli F., De Battista H., Vehí J. (2013). Postprandial blood glucose control using a hybrid adaptive PD controller with insulin-on-board limitation. *Biomedical Signal Processing and Control*.

[26] Rossetti P., Quirós C., Moscardó V. (2017). Closed-loop control of postprandial glycemia using an insulin-on-board limitation through continuous action on glucose target. *Diabetes Technology & Therapeutics*.

[27] Man C. D., Micheletto F., Lv D., Breton M., Kovatchev B., Cobelli C. (2014). The UVA/PADOVA type 1 diabetes simulator. *Journal of Diabetes Science and Technology*.

[28] Steil G. M., Palerm C. C., Kurtz N. (2011). The effect of insulin feedback on closed loop glucose control. *The Journal of Clinical Endocrinology & Metabolism*.

[29] Sala-Mira I., Díez J. L., Bondia J. (2017). Insulin limitation in the artificial pancreas by sliding mode reference conditioning and insulin feedback: an in silico comparison. *IFAC-PapersOnLine*.

[30] Wilinska M. E., Chassin L. J., Schaller H. C., Schaupp L., Pieber T. R., Hovorka R. (2005). Insulin kinetics in type-1 diabetes: continuous and bolus delivery of rapid acting insulin. *IEEE Transactions on Biomedical Engineering*.

[31] Brazeau A. S., Mircescu H., Desjardins K. (2013). Carbohydrate counting accuracy and blood glucose variability in adults with type 1 diabetes. *Diabetes Research and Clinical Practice*.

[32] Herrero P., Bondia J., Adewuyi O. (2017). Enhancing automatic closed-loop glucose control in type 1 diabetes with an adaptive meal bolus calculator-in silico evaluation under intra-day variability. *Computer Methods and Programs in Biomedicine*.

[33] Dalla Man C., Rizza R. A., Cobelli C. (2007). Meal simulation model of the glucose-insulin system. *IEEE Transactions on Biomedical Engineering*.

[34] Agiostratidou G., Anhalt H., Ball D. (2017). Standardizing clinically meaningful outcome measures beyond HbA1cfor type 1 diabetes: a consensus report of the american association of clinical endocrinologists, the american association of diabetes educators, the american diabetes association, the endocrine society, JDRF international, the leona m. and harry b. helmsley charitable trust, the pediatric endocrine society, and the t1d exchange. *Diabetes Care*.

[35] American Diabetes Association (2018). Glycemic targets: standards of medical care in diabetes—2018. *Diabetes Care*.

[36] Bergenstal R. M., Beck R. W., Close K. L. (2018). Glucose management indicator (GMI): a new term for estimating A1C from continuous glucose monitoring. *Diabetes Care*.

[37] Magni L., Raimondo D. M., Man C. D. (2008). Evaluating the efficacy of closed-loop glucose regulation via control-variability grid analysis. *Journal of Diabetes Science and Technology*.

[38] Ketema E. B., Kibret K. T. (2015). Correlation of fasting and postprandial plasma glucose with HbA1c in assessing glycemic control; systematic review and meta-analysis. *Archives of Public Health*.

[39] Bertachi A., Beneyto A., Ramkissoon C. M., Vehí J. (2018). Assessment of mitigation methods to reduce the risk of hypoglycemia for announced exercise in a uni-hormonal artificial pancreas. *Diabetes Technology & Therapeutics*.

[40] Ramkissoon C. M., Bertachi A., Beneyto A., Bondia J., Vehi J. (2019). Detection and control of unannounced exercise in the artificial pancreas without additional physiological signals. *IEEE Journal of Biomedical and Health Informatics*.

